The article "Ultrasound Image Texture Feature Learning-Based Breast Cancer Benign and Malignant Classification" was published in 2021. Journal: Comput Math Methods Med.

# Ultrasound Image Texture Feature Learning-Based Breast Cancer Benign and Malignant Classification

**DOI:** 10.1155/2021/6261032

**Published:** 2021-12-28

**Authors:** Huiling Gong, Mengjia Qian, Gaofeng Pan, Bin Hu

**Affiliations:** ^1^Department of Ultrasound, Minhang Hospital, Fudan University, Shanghai, China; ^2^Ruijin Hospital Affiliated to the Shanghai Jiao Tong University Medical School, Shanghai 200020, China; ^3^Department of Surgical, Minhang Hospital, Fudan University, Shanghai, China

## Abstract

The use of ultrasound images to acquire breast cancer diagnosis information without invasion can reduce the physical and psychological pain of breast cancer patients and is of great significance for the diagnosis and treatment of breast cancer. There are some differences in the texture of breast cancer between benign and malignant cases. Therefore, this paper proposes an adaptive learning method based on ultrasonic image texture features to identify breast cancer. Specifically, firstly, we used dictionary learning and sparse representation to learn the ultrasonic image texture dictionary of benign and malignant cases, respectively, and then used the combination of the two dictionaries to represent the test image to obtain the texture distribution characteristics of the test image under the two dictionary representations, which called the sparse representation coefficient. Finally, these above features were filtered by sparse representation and sent to sparse representation classifier to establish benign and malignant classification model. 128 cases were randomly divided into training and testing sets according to 2: 1 for training and testing. The proposed method has achieved state-of-the-art results, with an accuracy of 0.9070 and the area under the receiver operating characteristic curve of 0.9459. The results demonstrate that the proposed method has the potential to be used in the clinical diagnosis of benign and malignant breast cancer.

## 1. Introduction

Breast cancer is a serious threat to women's health and is one of the most common malignant tumors in women all over the world. According to the latest prediction of the “Clinician Cancer Journal” [1], in 2018, among about 879,000 new cancer cases in American women, there were 266,000 cases of breast cancer, accounting for about 30.26% of all female cancer cases, with the highest incidence rate. Among the approximately 286,000 female cancer deaths in the United States, breast cancer is approximately 41,000, accounting for approximately 14.33% of all female cancer deaths, and the death rate ranks second. Early detection, early diagnosis, and early treatment of breast cancer are the keys to increasing the cure rate and improving the prognosis.

At present, the clinical methods of breast tumor detection mainly include palpation, puncture, and medical imaging technology. The medical imaging techniques used on breast tumors are mainly ultrasound imaging, mammography, and magnetic resonance imaging. Compared with other commonly used methods of breast tumor detection, the main advantages of ultrasound imaging are simple and convenient operation; noninvasive and no harm to the human body; no radiation, safe, and reliable; high real-time, fast imaging, facilitate the specific patient to do targeted examination; and low prices, suitable for large-scale promotion [2, 3]. It is of great significance to the clinical diagnosis and treatment of breast cancer to explore the deep pathological features of breast ultrasound images and obtain the results of benign and malignant tumors noninvasively.

In the past ten years, with the development of pattern recognition tools and the expansion of data sets, the use of engineering image processing technology to diagnose medical diseases has become a new trend. These advances have promoted the development of the high-throughput extraction process of quantitative features and led to the conversion of images to high-dimensional data features and subsequent decision support using these data. This approach is called radiomics [3]. The combination of high-dimensional data features of radiomics and other patient data can further improve the accuracy of diagnosis and prognosis. In 2014, an article published in the journal *Nature* proposed the use of high-throughput features of images for tumor subtype identification [4], and then, some researchers have proposed using high-throughput features to predict tumor molecular markers [5] and tumor classification and achieved better results.

Sparse representation theory believes that natural signals can be formed by linear combinations of a few atoms in the dictionary, and these atoms contain the most essential characteristics of the signal [6]. The advantages of sparse representation in signal expression analysis make it widely used in the fields of data compression, signal denoising, signal separation, image restoration, classification, and recognition. A dictionary is used to sparsely represent the noisy image or signal and then reconstruct the representation coefficients to get the denoised image or signal. In the classification and recognition problem, the characteristics of the test sample are represented by the known label features, and then, the residual comparison can accurately predict the sample category to be tested [7]. Li et al. [8] use the sample feature to sparsely represent the sample label, and according to the obtained sparse representation coefficient, the sample features are ranked by importance, and the biomarker features of schizophrenia are effectively selected. Sparse representation has the advantages of image and data expression analysis, making it an important tool for image segmentation, feature extraction, feature selection, and classification discrimination in radiomics.

Previous clinical literature reports that there are many differences in the imaging morphology of benign and malignant breast cancer cases, such as orientation, margins, calcification, and internal echo. These differences are reflected in the differences in the texture details of the images. Therefore, inspired by the idea of radiomics and combined with the theoretical basis of sparse representation, this paper proposes a method for identifying benign and malignant breast cancer based on the learning of ultrasound image texture features. To extract the texture features of the tumor area, we firstly trained the texture feature dictionary, then used the dictionary to sparsely represent the set of image patches, which are extracted from the test sample tumor area; finally, the sparse representation coefficients of all image patches are averaged to obtain the texture features corresponding to each tumor sample. Because the directly extracted texture features have a certain degree of redundancy, an iterative sparse representation method is established to select a few features with high stability and high resolution, and the iterative solution process effectively overcomes the lack of training samples and the inefficient use of training sample information during feature selection. Finally, the sparse representation method is used to classify and identify the selected tumor features.

## 2. Method

### 2.1. Image Segmentation

The segmentation of the tumor region is the premise and basis for subsequent feature extraction and classification and recognition. We ask two experienced doctors to mark the lesion area, one for segmentation and the other for verification.  Figure 1 shows the segmentation results of two cases. Benign cases on the left and malignant cases on the right. The area within the white curve is the focus area.

### 2.2. Feature Extraction of Texture

Due to the large differences in the size and shape of tumors in different patients, image patch-based processing methods are used to extract tumor texture features.  Figure 2 shows the flow chart of image texture feature extraction based on sparse representation. First, extract the image patch set of the tumor area *P* ∈ *R*^*n*×*N*^, *P* = [*p*_1_, *p*_2_ ⋯ *p*_*N*_], *p*_*i*_ represents the *i*-th image patch, and *N* is the number of image patches contained in the tumor area. Multiple benign image patch sets and multiple malignant image patch sets were selected, respectively, and *k*-singular value decomposition (KSVD) is adopted to train the benign dictionary *D*_*B*_ ∈ *R*^*n*×*K*^ and the malignant dictionary *D*_*M*_ ∈ *R*^*n*×*K*^ [6], and the training dictionary is combined to obtain the texture feature extraction dictionary *D* = [*D*_*B*_, *D*_*M*_] ∈ *R*^*n*×2*K*^.  Figure 3 shows the trained benign dictionary and malignant dictionary.

The atoms in the dictionary, that is, the small square area enclosed by the blue line in Figure 3, represent the tiny texture details of the image, and the tumor image is composed of these small details superimposed. Comparing the two dictionaries, it is obvious that the texture details which make up the benign image and the texture details that make up the malignant image are quite different. Therefore, an intuitive idea to distinguish between benign and malignant is to use the atoms (textures) in the dictionary to express the image to be detected and compare the statistical differences of atoms used to constitute the images to be detected to identify tumors, that is, to use the dictionary to perform sparse representation of detected tumor images, and then, sparse representation coefficients (descriptions of texture information used to constitute tumor regions) are used as the corresponding feature and subsequently sent to classifiers as an input to identify tumors.

For the tumor area to be detected, a dictionary *D* is used to sparsely represent its corresponding image patch set *P*.

(1) $$\begin{array}{c} \hat{\Lambda }=\underset{\Lambda }{\text{argmin}}{\left\|P-D\Lambda \right\|}_{2}^{2}+\rho \phi \left(\Lambda \right). \end{array}$$

Among them, *Λ* = [*α*_1_, *α*_2_, ⋯, *α*_*N*_], *α*_*i*_ ∈ *R*^2*K*^ is the corresponding sparse representation coefficient corresponding to *p*_*i*_, *ϕ*(·) is the sparse constraint function, and *ρ* is the weight control parameter. Because the number of image patches extracted from different tumors is different, the corresponding *Λ* size is different, which is not conducive to the subsequent design of the classifier. Therefore, the image patches in the image patch set are individually sparsely represented, and the absolute value of the sparse representation coefficient is averaged as the texture feature of the tumor. Orthogonal matching pursuit (OMP) algorithm can quickly and effectively solve the sparse representation model in Equation (1).

Figures 4(a) and 4(b) are the texture features of benign and malignant, respectively, showing obvious differences between them. The first half of benign feature (1 ~ 900, corresponding to benign dictionary) is generally larger than the second (901~1800, corresponding to benign dictionary), while the malignant characteristic situation is the opposite. That is, as shown in Figure 3, benign images are more represented by textures in the benign dictionary, and malignant images are more represented by atoms in the malignant dictionary. In addition, as shown in Figure 4(a), benign uses the most frequently texture information (feature coefficients pointed to by the yellow arrow) from the benign dictionary, while in Figure 4(b), malignant uses the most texture information (feature coefficients pointed to by the red arrow) from the malignant dictionary. It can be seen that there are obvious differences between the two. Therefore, the statistical distribution difference of the two kinds of tumor texture information is of key significance for tumor identification.

In addition to texture features, previous studies have found that benign and malignant tumors are related to morphology and gray level. Therefore, we further extract 33 features describing tumor shape and gray level, as shown in Table 1, including 18 gray level features and 15 shape features. And in the experiment, we compared the classification results using only texture features with the classification results integrating texture, gray level, and shape features.

### 2.3. Feature Selection Based on Sparse Representation

There is a large amount of redundant information in the texture features. These redundant features not only increase the calculation amount of subsequent classification and recognition but may also affect the recognition accuracy. Therefore, a sparse representation feature selection model is established to select a small number of high-resolution features.

(2) $$\begin{array}{c} \hat{w}=\underset{w}{\text{argmin}}{\left\|y-Fw\right\|}_{2}^{2}+\gamma {\left\|w\right\|}_{0}, \end{array}$$

where *y* ∈ *R*^*m*^ is the training sample label, *m* is the number of training samples, *F* = [*f*_1_, *f*_2_ ⋯ *f*_*m*_]^*T*^ ∈ *R*^*m*×2*K*^ is the training sample feature set, and *γ* is the sparse representation of the control parameter and sparsely represents the importance of the feature corresponding to the absolute value of the element in the coefficient *w*. While *w* is obtained, the key features can be selected through a simple threshold comparison.

It is worth noting that in the actual feature selection, the number of samples *m* will have an important impact on the selection results. On the one hand, when *m* < <2*K*, the effective sparse coefficient solution can be obtained by solving Equation (2); however, due to the small number of samples, the sparse representation coefficients obtained by an iterative solution cannot reflect the importance of some features well; on the other hand, when *m* > 2*K*, Equation (2) is not suitable for the overdetermined problem at this time. In addition, for the feature selection of Equation (2), the performance of feature selection should increase with the increase of the number of samples.

Iterative sparse representation feature selection method effectively solves the problem of the number of samples in feature selection. In each iteration, *M* < <2*K* samples are randomly selected from the sample set for sparse representation, which ensures the effectiveness of the sparse solution in Equation (2). In addition, the data in the sample set is randomly selected multiple times for sparseness, and the obtained coefficients are averaged, which not only the information of all sample data is utilized but also the robustness of sparse solution is increased, and the validity of selection feature is guaranteed.  Figure 5 shows the change of residuals represented by features to sample labels as the number of samples increases after features are sorted by sparse representation. It can be seen that only the first 300 features have a significant representation effect on labels among the extracted features.

In fact, the essence of sparse representation feature selection is to select a few features with high correlation with sample tags, and when OMP algorithm is used to solve Equation (2), the orthogonalization process eliminates the redundancy among the selected features, so the final selected features meet the characteristics of maximum correlation and minimum redundancy.

### 2.4. Sparse Representation-Based Classification (SRC)

For the screened features, the SRC method [7] is used for classification verification. Suppose **F** = [**F**_1_ ⋯ **F**_**c**_ ⋯ **F**_**C**_] denotes the feature set of training samples from **C** classes, **F** represents the feature selection result of **F**, and **F**_**c**_ is the sample feature set of class *c*. The dictionary learning method is aimed at learning some discriminative dictionaries from **F**, whose model can be formulated as [9].

(3) $$\begin{array}{c} \left\{\Psi ,\Phi \right\}=\underset{\Phi ,\Psi }{\text{argmin}}\overset{C}{\underset{c-1}{\sum }}{\left\|F_{c}-\Psi_{c}\Phi_{c}F_{c}\;\right\|}_{F}^{2}+\lambda {\left\|\Phi_{c}\bar{F_{c}}\right\|}_{F}^{2},\text{s}.\text{t}.{\left\|\varphi_{q}\right\|}_{2}^{2}\leq 1, \end{array}$$

where is *λ* a scalar constant and $\bar{F_{c}}$ is the complementary matrix of **F**_**c**_ in the whole feature **F**. Dictionary pair Ψ = [Ψ_1_ ⋯ Ψ_**c**_ ⋯ Ψ_**C**_] is used to reconstruct and code **F**, respectively. *φ*_*q*_ is an atom of dictionary Ψ. When the dictionary pairs Ψ and **Φ** are learned, the classification model can be formulated as:

(4) $$\begin{array}{c} l_{l}=\underset{c}{\text{argmin}}{\left\|f_{l}-\Psi_{c}\Phi_{c}f_{l}\right\|}_{2},c\in \left[1,\cdots ,C\right]. \end{array}$$

## 3. Experimental Results

The data of 128 cases were used for retrospective study, of which 61 cases were benign and 67 cases were malignant. The size of the ultrasonic image is 910∗630. The data set was randomly divided into training and testing according to 2 : 1, including 85 training sets and 43 testing sets. The training set is used for texture dictionary training, feature screening, and classification model establishment. When the model is established, the test data were begun to testing directly. We used accuracy (Acc), sensitivity (Sen), specificity (Spe), positive predictive value (Ppv), negative predictive value (Npv), and area under the receiver operating characteristic (ROC) curve (Auc) to evaluate the classification results of the model [10]. In which, Sen represents the ratio of the number of correctly discriminated benign cases to the total number of benign cases, and Spe represents the ratio of the number of correctly discriminated malignant cases to the total number of malignant cases.

In this method, the image patch size is 15∗15, the sliding distance of the extracted image patch is 7∗7, and the size of the training benign and malignant dictionaries is 225∗900. Therefore, the dictionary *D* size is 225∗1800, and the number of corresponding extracted features is 1800. In the process of feature selection, *ε*, *K*_0_, and *M* are set as  *ε* = 0.0001, *K*_0_ = 300, and *M* = 5, respectively. The coefficients in SRC are norm constrained by *l*_*p*_ = 0.5.

We compared the classification performance of texture features only using adaptive learning and features combining texture, gray, and shape. The results are shown in Table 2. In the table, we can see that the two methods have achieved excellent performance, and the classification accuracy has reached 0.8837 (texture feature only) and 0.9070 (combined features). This shows that our self-adaptive learning-based texture features can effectively distinguish breast cancer from benign and malignant. Multifeature combination method is better than the texture feature only. It shows that the shape and grayscale features of breast cancer ultrasound images play a certain role in differentiating benign and malignant tumors.  Figure 6 shows the ROC curve of the classification results of the two comparison methods. It can be seen from the indicators such as Sen and Spe in the classification curve and table that the proposed method not only has high classification accuracy but also the proportion of misjudgment of positive and negative samples is relatively similar, so it has high clinical applicability.

## 4. Discussion

Early detection and diagnosis of breast cancer is an effective way to improve the cure rate of breast cancer patients and reduce the mortality rate [11–13]. One of the most important indicators for early diagnosis is to determine the benign and malignant lesions. Ultrasound images are easy to find the location of breast lesions, but it is difficult to distinguish benign and malignant tumors from images, and the diagnostic accuracy is limited. Histopathological diagnosis is the gold standard for the diagnosis of benign and malignant breast cancer. However, needle biopsy is invasive and can bring physical pain and mental anxiety to the patient [14]. Based on ultrasound images, we use medical image data mining methods to noninvasively obtain diagnostic information of benign and malignant. As reported in the past, ultrasound images of benign and malignant breast cancer have differences in structure and texture. Therefore, we propose an adaptive texture feature learning method to extract discriminative texture features and then use the sparse representation system for feature screening and classification recognition.

Some traditional radiomics methods design manual features based on clinical experience to build machine learning classification models [15]. However, due to the limitations of existing clinical experience, some deeper-level and move discriminative features are often difficult to effectively mine and quantify. In contrast, our proposed image texture feature extraction method based on adaptive learning can automatically extract and quantify the inherent texture structure information of different types of images through dictionary training (as shown in Figure 4), which improves the effectiveness of features and the robustness of models.

Feature selection is a key step in building a machine learning classification model, because selecting a few more discriminative features can reduce the risk of model overfitting and the model computational complexity. The *t*-test *P* value comparison is a commonly used feature selection method for radiomics models, but this method can only evaluate the importance of each feature individually, ignoring the impact of feature combination on the performance of the classification model. This paper uses the sparse representation method for feature selection. In the process of feature selection, both the correlation between features and class labels, and the redundancy between features are considered, which is conducive to selecting the optimal feature subset.  Figure 7 shows how the model classification accuracy changes with the increase of feature number in the feature set. It can be clearly seen that the classification accuracy increases with the increase in the feature number within a certain range.

Table 3 and Figure 8 show the classification results of different classifiers in the same feature subset. The SRC in our model is better than support vector machine (SVM) and Adaboost on the whole, and the accuracy of classification results is improved by more than 5%. This is because, for small sample classification problems, nonparametric training-based SRC can better inhibit model overfitting than parameter training-based SVM and Adaboost.

Although in our experiment, we strictly divide the training set and the test set, the stability and reliability of the model need to be further verified on a variety of breast cancer data. Therefore, in future work, we will collect multicenter data and then train and test on different center data sets.

## 5. Conclusion

In order to noninvasively obtain diagnostic information of benign and malignant breast cancer from ultrasound images, we first proposed a dictionary training-based method to adaptively extract different texture features of different types of tumors and then use the sparse representation method for feature selection and classification. A retrospective study of 128 cases of data shows that the method has achieved encouraging performance with a classification accuracy of 0.9070. The proposed method may be used for clinical diagnosis of benign and malignant breast cancer, thereby improving the efficiency of breast cancer diagnosis and reducing patient suffering.

## Figures and Tables

**Figure 1:** The segmentation results are shown. Benign cases on the left side and malignant cases on the right side. The area within the white curve is the focus area.

**Figure 2:** The flow chart of image texture feature extraction based on sparse representation.

**Figure 3:** The trained dictionary.

**Figure 4:** The extracted texture feature: (a) benign texture feature; (b) malignant texture feature.

**Figure 5:** Iterative convergence curves of residual.

**Figure 6:** The ROC curves of the two methods. (a) The ROC curve of the texture feature-based classification. (b) The ROC curve of the combined feature-based classification.

**Figure 7:** The classification accuracy varies with the number of features.

**Figure 8:** The ROC curves of different methods.

**Table 1:** Summary of 33 features.

Feature category	Feature name	Feature number
Intensity	(1) Energy; (2) h-entropy; (3) kurtosis; (4) max; (5) mean absolute deviation; (6) mean; (7) media; (8) min; (9) range; (10) root mean square; (11) skewness; (12) standard-deviation; (13) h-uniformity; (14) variance; (15) h-mean; (16) h-variance; (17) h-skewness; (18) h-kurtosis	18
Shape	(1) Compactness; (2) compactness-square; (3) max-length; (4) spherical disproportion; (5) sphericity; (6) superficial-area; (7) surface to volume ratio; (8) volume; (9) region to bounding-box ratio; (10) max major-length; (11) min minor-length; (12) eccentricity; (13) orientation; (14) solidity; (15) Fourier-descriptors	15

**Table 2:** Comparison of classification results of different methods.

Methods	Auc	Acc	Sen	Spe	Ppv	Npv
Texture feature	0.8810	0.8837	0.8636	0.9048	0.9048	0.8636
Combined feature	0.9459	0.9070	0.9091	0.9048	0.9091	0.9048

**Table 3:** Comparison of classification results of different classifiers.

Methods	Auc	Acc	Sen	Spe	Ppv	Npv
SRC	0.9459	0.9070	0.9091	0.9048	0.9091	0.9048
SVM	0.8874	0.8140	0.7273	0.9048	0.8889	0.7600
Adaboost	0.9026	0.8372	0.7727	0.9048	0.8947	0.7917

## Data Availability

The datasets used and/or analyzed during the current study are available from the corresponding author on reasonable request.
